# Implementing Critical Machine Learning (ML) Approaches for Generating Robust Discriminative Neuroimaging Representations Using Structural Equation Model (SEM)

This article has been retracted.

**DOI:** 10.1155/2022/6501975

**Published:** 2022-04-14

**Authors:** Mohammed Rashad Baker, D. Lakshmi Padmaja, R. Puviarasi, Suman Mann, Jeidy Panduro-Ramirez, Mohit Tiwari, Issah Abubakari Samori

**Affiliations:** ^1^Department of Computer Techniques Engineering, College of Information Technology, Imam Ja'afar Al-Sadiq University, Baghdad, Iraq; ^2^Department of Information Technology, Anurag University, Hyderabad, Telangana State, India; ^3^Saveetha School of Engineering, Saveetha Institute of Medical and Technical Sciences, Chennai, Tamil Nadu, India; ^4^Information Technology Department, Maharaja Surajmal Institute of Technology, New Delhi, India; ^5^Business Department, Universidad Tecnológica del Peru, Peru; ^6^Department of Computer Science and Engineering, Bharati Vidyapeeth's College of Engineering, A-4, Rohtak Road, Paschim Vihar, Delhi, India; ^7^School of Engineering Sciences, University of Ghana, Ghana

## Abstract

Critical ML or CML is a critical approach development of the standard ML (SML) procedure. Conventional ML (ML) is being used in radiology departments where complex neuroimages are discriminated using ML technology. Radiologists and researchers found that sole decision by the ML algorithms is not accurate enough to implement the treatment procedure. Thus, an intelligent decision is required further by the radiologists after evaluating the ML outcomes. The current research is based on the critical ML, where radiologists' critical thinking ability, IQ (intelligence quotient), and experience in radiology have been examined to understand how these factors affect the accuracy of neuroimaging discrimination. A primary quantitative survey has been carried out, and the data were analysed in IBM SPSS. The results showed that experience in works has a positive impact on neuroimaging discrimination accuracy. IQ and trained ML are also responsible for improving the accuracy as well. Thus, radiologists with more experience in that field are able to improve the discriminative and diagnostic capability of CML.

## 1. Introduction

Neuroimaging discrimination through the use of ML approaches has seen a positive demand in the modern world. However, this trending feature can effectively generate different robust as well as discriminative neuroimaging representations by radiologists. In order to strengthen the abilities of discrimination, critical ML approaches have seen a positive growth towards acquiring more accurate recognizing and evaluating images. Today, in various medical and healthcare areas, ML is broadly utilized for recognizing as well as generating various neuroimaging materials [1]. With the help of different stages and phases in ML, the tendency towards generating three-dimensional neuroimages has reflected significant advantages in clinical aspects. On the other hand, various pieces of evidence shed some important lights on remote sensing of medical images and their recognition. Through the use of ML approaches, it has become more relevant for the development of human health in the sustainable future. Researchers have identified algorithms for generating robust and discriminative neuroimages through ML approaches. Moreover, the application analysis through the use of the “structural equation model” will be highly beneficial for conducting the entire research study.  Figure 1 shows the flowchart of the generation of neuroimages.

On the other hand, the utilization of ML has seen relevant growth in the modern-day medical aspects. For investigating more accurately various neurological as well as psychiatric disorders worldwide, ML approaches can be greatly used. It can also be used for predicting and analysing numerous health-related outcomes [2]. However, by using the SEM model, this analysis can be easily conducted by manipulating different predictions of functions. In contrast to that, different nonlinear and linear predictions can also be delivered by a simple procedure for implementing inference strategies and theories. Neurological computers can process ML methods in order to align all the kernel-transformed native features of engineered input vacuums [3].

The basic purpose of the study is to investigate the implementation of critical ML (ML) approaches for generating robust discriminative neuroimaging representations; these applications of new and innovative tools support the enhancement of the neuroimaging aspects in the industry. Furthermore, the study is intended to use critical statistical tools which enable in addressing the needs of implementing these methods in an efficient manner. The trend to create 3D neuroimaging across different stages and phases of ML reflects significant clinical benefits. On the other hand, the various elements significantly illuminate remote analysis and recognition of medical images. Through the application of ML methods, it has become more important for the future sustainable development of human health.

This process can at once help in generating robust as well as discriminative neuroimages by modelling the patients' data in their brains. An effective boosting technique also can be applied in the SEM model analysis process to enhance the performance of ML approaches. In order to recognize and create important neuroimages, a discriminative and robust approach has been undertaken in order to mitigate all the invalid input space. Through applying features from an expert-designed variables' subset, relevant clinical data and images can be effectively recorded by ML methods for further investigation.  Figure 2 shows the graph that reflects the generation of neuroimages through machine learning.

Today, representing and generating neuroimaging techniques can function at a deeper level in medical science by using ML approaches. However, by using this technique, different anatomical activities of patients' brains can be determined by generating valid neuroimages. On the other hand, ML methods are also necessary for measuring the brain structures' integrity as well as their internal functions and connections. By producing discriminative neuroimages from a robust perspective, all the chemical, psychological, metabolic, and electrical impulses in brain functions can be effectively diagnosed [4]. Therefore, the researchers have identified the critical ML technique to improve the accuracy of standard ML technique. Due to the complex image formation by scanning, the ML devices cannot accurately diagnose and determine the treatment procedures. Thus, critical thinking and evaluation is required by the researchers to improve neuroimaging discrimination accuracy.

Previous studies conducted in the area of study are more focused in creating algorithms and contemplating on models which will enhance on neuroimaging; however, very few studies were focused in making critical statistical analysis in order to validate the model and present the information in an efficient manner; hence, the research gap of applying statistical models were highly limited in the ML-based neuroimaging approached; therefore, the researcher has intended to prepare the article which enable in implementing critical ML approaches in neuroimaging.

## 2. Literature Review

Medical science nowadays has experienced a positive impact of ML approaches in clinical progression, image generation, and classification. The robust and discriminative neuroimage processing has become more efficient through the use of different ML approaches. This critical ML approach with the SEM model is beneficial for generating important neurological images that need to be analysed from a positive perspective. In order to understand the functions of the brains, it has been observed that all the uses of ML algorithms are highly essential for generating relevant neuroimages [5]. This overall method can be effectively conducted by implementing neural network settings in a convolutional manner. However, different clinical methods for generating neuroimages through ML approaches provide beneficial representations by determining relevant boundaries of the decision in various healthcare aspects. There can be traced various innovative applications of ML in clinical as well as technical aspects of neurological imaging. Moreover, ML uses the strategies of artificial neural network setting. With the help of this architecture, image resemblance to the neurological diseases of human can be effectively conducted through different cognitive functions.

After analysing all the impacts of ML, the convolutional layers have been seen to have a strong connection with generating robust neuroimages in the size of little squares. The process of generating as well as recognizing discriminative neuroimages can be analysed by physicians with the use of ML learning through part-by-part evaluation. On the contrary, necessary brain function input spaces related to a clinical image have been correlated with the ML stages. Towards investigating its amplified growth across various clinical channels worldwide, an efficient application of ML methods is highly considerable [6]. However, functional neuroimages related to the brain contain noisy as well as more complex information that can be effectively captured by using ML learning. This process using the SEM model would be easy to understand for the researchers and physicians while investigating neural indirect signatures. Under the cognition methods of any experimental medical structure, this approach finds its way better to analyse medical images. Those algorithms used in the ML system can be highly used in the neurological science. On the contrary, it can generate the best features of discriminative robust neuroimages in order to understand and diagnose serious neurological disorders globally [7].

Neuroimaging is a process of brain imaging found in modern clinical aspects across the globe that can be recognized through the use of proper ML approaches. However, by using various ML techniques, brain function images can be effectively generated. These images are at once essential for both the physicians and staff of hospitals in order to identify and diagnose various brain functions. Along with this, this approach also helps in detecting brain structural issues, symptoms of pharmacology, and numerous problems of the nervous system [8]. After analysing and generating these images through the use of proper ML learning methods, physicians can successfully invent and implement numerous treatment methods with neuroscience medicines. In order to overcome and understand various psychological issues, generating robust and discriminative neuroimages can at once provide necessary benefits to the modern clinical fields. On the other hand, with using relevant ML approaches, various functions of brain circuits in the clinical lobe of temporal order can be effectively observed. Recently, AI technologies are being vastly used by ML researchers in order to facilitate effective methods of implementing episodic memory devices. Analysing these ML algorithms can offer an easy understanding of the complex psychological issues regarding proper episodic control.  Figure 3 shows the generation of neuroimages with the help of machine learning approaches.

In contrast to that, it has been observed that ML approaches allow researchers to identify numerous statistical patterns from a vast set of data. However, generating neuroimages from a discriminative and robust perspective has several benefits in the clinical aspects. In order to solve various issues related to broad tasks in the healthcare sector, neuroscience has adopted the strategies of the ML processes. On the other hand, these efficient methods can automate the valid evaluation of vast amounts of clinical datasets related to neuroscience. However, by using the methods of deep network processes, physicians can effectively gain relevant insight into the learning and functions of the brain and psychology of patients [10]. Today, a large variety of ML approaches are being used in medical sectors for detecting and generating relevant images towards further diagnosis and providing necessary treatments. The ML technology can also be used for generating as well as evaluating neurological images from clinical aspects. On the contrary, the robust and discriminative generation of neuroimages also reflects excellent performance in ML applications, registration, and psychological segmentation. Moreover, the robust process of neuroimage generation can be effectively done by the physicians towards calculating various ML mathematical algorithms.

On the other hand, ML approaches in the healthcare sector can also offer the necessary digital diagnosis of various neurological and psychological disorders. One of the most essential reasons behind applying ML learning approaches for generating neuroimages is that it can detect symptoms and patterns of several diseases. On the contrary, the learning methods also help physicians to determine proper information from the electronic healthcare records of a patient. However, while detecting any anomalies within the neurological system, ML learning provides tremendous aid in generating relevant images. Physicians also tend to apply these important methods for demonstrating the results of neuroimages to the patients. It has been observed that ML learning can proactively detect and recognize possible pathways of neurological disease as well as their outcomes regarding various beneficial scopes for treatments [11]. Moreover, by generating those necessary clinical images, ML can at once improve the efficiency of the overall hospitals as well as health systems in a cost-efficient way.  Figure 4 shows the treatment of neurological diseases with the help of machine learning.

The modern-day medical system has seen beneficial utilization of ML approaches in both generating and detecting various images, especially neurological reflections. A broad range of ML applications can be highly used for generating neurological images by enhancing the opportunities for clinical improvements soon. Besides, efficient handling and diagnosis of those images also can be conducted by the ML procedures following the functions of neural network systems. Proper selection and analysis of ML algorithms make it easy for physicians to use this method for generating images regarding neurological as well as psychological factors [12]. On the contrary, the particular method can be conducted efficiently by the implementation of relevant algorithms as well as information regarding patients' information automation.

ML in today's medical world helps in gathering patient insights as well as learning through creating scopes for more neurological treatments. All these opportunities in the clinical sectors at once lead the entire research towards a predictive analysis related to the particular topic. Quickly acquiring brain functions' insights provides necessary aid to the neurological diagnosis in order to detect major aspects of a patient. Moreover, by utilizing the ML approaches, detection and generation of relevant medical images can be improved in the future for serving patients in a better way. ML approaches mainly include AI data subset especially designed for generating discriminative and robust patterns of neuroimaging representation. Due to the need for better analysis of neuroimages for the sake of improving the diagnostic process, the integration of ML occurred in the early 2000s. As a consequence of this, the ability of neuroimaging studies in the context of mapping the brain function and brain structure of an individual has improved significantly.

The method of support vector machine (SVM) has improved the general interpretation of the learned model. This method is based on the principles which are developed for minimizing the structural risk factors. The method of SVM was popular in the field of neuroimaging studies in the late 1990s. The versatile feature of SVM which enables an individual to use this method in different types of the kernel has increased its popularity [13]. Moreover, the capability of SVM to cope with nonlinear boundaries using the method of kernel mapping made it extremely robust in this field. Another popular method that attracted the focus of neuroimaging studies in the period of early 2000s was random forests. The rigorous research over approximately ten years on ensemble was mainly accountable for the emergence of this method. The main aspect of the ensemble is to decrease the flaws of a method. Ensembles mainly use several models and select random features from this model to minimize the errors. This aspect of the ensemble makes it a pivotal player in neuroimaging studies. Besides, they do possess impactful generalization characteristics, and their power to cut down the noise to promote the true signal is also immensely versatile. The relevance of ensembles is still enormous as they are now used in parallel to deep learning for the improvement of the neuroimaging process.

Deep learning is the most recent development that has taken place in this field. The future of deep learning seems to be extremely promising in the context of neuroimaging studies for its several positive traits. The ability of deep learning networks to learn the complex aspects of neuroimaging sequentially is extremely critical. In addition, deep learning networks are highly adequate to construct nonlinear boundaries [14]. Also, there is a negligible amount of chance for mishaps regarding data overfit and generalization of new data and models. The only chance for a deep learning network to produce a false output is when a large amount of data are given to it for its training. Mostly in this sort of case, a significant time lag, as well as falsified output, is noticed. In this sort of case, a deep learning network often takes the assistance of ensembles to minimize its gaps.

Deep learning is significantly improved over the years by the incorporation of structural equation models (SME) [15]. The segments like the processing of images, classification for diagnostic, linear as well as nonlinear regression, characterization of diseases, and prediction of diseases have seen enormous success in the recent days by the introduction of deep learning. The success of deep learning has increased up to that much extent that the expectation is sometimes going beyond its proportion. There is already hype going on in the field of neuroscience due to its ability to visualize and learn complex properties of the brain and nervous system. For the simplification of these complexities, often scientists are in favour of integrating deep learning with structural equation models. However, the integration and implementation of these two are limited to certain aspects of neuroimaging studies, and better ways of fusion are needed for the enhancement of neuroscience in the recent future. The plot of fitting of brain-age regressor of a community of aging people is shown in Figure 5.

The relevance and advantages of using these methods in neuroimaging studies are quite significant in the present circumstances. Numerous disorders and diseases can be diagnosed by using ML in the context of neuroimaging studies. Diseases like Alzheimer's, schizophrenia, and mood disorders can easily be detected by using ML nowadays. In parallel to that, brain aging and brain disorders can also be detected by using ML [16]. It is worth saying here that the future of diagnostics is largely dependent on the development of ML. The ML network can also be used in distinguishing people based on their fingerprints. Therefore, ML and its development can enhance the performance of cognitive neuroscience in the upcoming days.

The deep learning network is also taking the help of neural networks for improving its performance. These approaches are essential for classifying as well as generating various clinical images. With the help of these images, issues related to numerous neurotically as well as psychological aspects can be diagnosed. Some of these networks are expected to perform like a human and extension of their performance beyond the level of human performance is possible. The incorporation of conventional neural networks is proving to provide a sustainable contribution in the field of neuroimaging studies. As the traditional neural networks are inefficient to provide larger prospects in the context of scalability as well as bandwidth in neuroscience, therefore the incoming steps of the modern neural networks are of cardinal importance for the betterment of neuroimaging studies.

The literature review has identified the common deep learning (DL) and ML practises that are used in neuroimaging representation. However, the increase in accuracy of neuroimaging representation has not been identified in the previous literature. Therefore, the researchers have found a way to understand how certain factors impact the accuracy of neuroimaging representation. The standard ML and critical ML are probably two different approaches that have significant impacts on generating and discriminating robust neuroimaging representation. The CML is based upon critical thinking and more ML experiences which will develop the accuracy further [17]. Sambasivam and Opiyo found that an unbalanced dataset had a major negative impact on the image classification by ML. Therefore, critical ML is probably required for evaluating the outcome of the proposed result by ML. Otherwise, serious negative impacts may cause social violence [18].

## 3. Research Methodology

Primary quantitative methods have been followed in this research for collecting survey data. The survey has been carried out in a healthcare sector where neuroimaging is carried out by using ML, DL, and conventional radiology approaches. The conventional approaches include detecting and evaluating the MRI (magnetic resonance imaging) images by the professionals themselves where the ML and DL perform the evaluation without any professional. The healthcare sector has both experienced and inexperienced radiologists who perform MRIs. However, a significant gap might be present between experienced and inexperienced radiologists that can have an impact on neuroimaging accuracy. To understand the impact, a survey has been carried out to understand how experience in radiology affects neuroimaging accuracy. Apart from this, ML training, gender of the professionals, age, and ML training will be assessed for understanding the accuracy change in neuroimaging representation and discrimination. The descriptive design is used for the study as it enables rendering better insights into the subject area, the implementation of ML approaches in medical industry is gaining more importance in recent years, and hence, it is highly significant to use better design in understanding the subject area; quantitative tools are used for measuring and validating the data an present them in a critical manner.

A total of 20 respondents were selected in the healthcare sector who work as a radiologist. They were responsible for understanding the neuroimages generated from MRI scans. However, both experienced and inexperienced radiologists were present, who provided the answers to the survey questions. The survey questions and answers were collected in Microsoft Excel and analysed using IBM SPSS.

The researcher has carried out multiple regression techniques using dependent and independent variables via IBM SPSS software version 26. One dependent variable has been selected which is the *accuracy of critical ML*. Thereafter, how the independent variables impact the accuracy will be identified through multiple regression analysis. The independent variables selected are *age*, *gender*, *experience in radiology*, *years of training in radiology*, *training years provided to the ML algorithms*, and *IQ of the respondents*. The sample size here is 20 (*n* = 20) where 20 respondents were selected only. The survey was conducted online due to the pandemic situation where the respondents gave answers via a Google form. The responses were further analysed and interpreted by regression analysis.

After regression analysis and interpretation, the researcher has drawn the structural equation model (SEM) by using Microsoft Word. Due to a lack of access to the premium version of IBM AMOS software, the researcher has selected Microsoft Word for drawing SEM. The SEM model explains the impacts of independent variables on the dependent variable. The researcher has also found that the independent variables have an impact on the independent variables as well. Therefore, SEM modelling will be beneficial to understand how the independent variables affect the independent as well as the dependent variable.

The significance value below 0.05 (*p* < 0.05) has been considered significant, and a Pearson correlation value near ±1 has been considered a *strong correlation*. After interpreting the SPSS output data, secondary research has been accomplished to discuss the interpretation. Secondary data allows the researchers to understand other behavioural disciplines and results from other researchers [19]. Therefore, the secondary data along with primary findings allow a researcher to discuss the results more critically. Thus, secondary data were collected from available online journal articles belonging to the last 5 years (2018-2022), and the final discussion has been made.

## 4. Analysis and Interpretation

A total of 20 respondents were selected to understand how different independent variables impact the dependent variable. Moreover, how the independent variables impact the dependent variables has been analysed as well. The data output has been analysed at a confidence interval of 95% because the true value may extend to a false value at over 95% confidence interval [20].

The descriptive statistics in Table 1 shows that the average IQ of the respondents is 102.90. It suggests that radiologists have an above-average IQ of 102.9. The average IQ differs in different countries where the IQ ranges from 80 to 120 [21]. Therefore, an IQ over 100 has been considered a good IQ value for radiologists. Table 1 also shows that the mean training period provided to the ML in neuroimaging is 3.95 years. This suggests that the training to ML in neurologic imaging is provided for approximately 3.95 years. Table 1 also suggests that males are the dominating radiologists in the neuroimaging representations. The average mean age of workers who work in neuroimaging representation is 39 where the mean accuracy belongs to 95.885%. However, the standard deviation in age is significantly higher which suggests people of different age groups belong to the radiology department. Concerning this, Figure 3 suggests that the age group varies significantly among the radiology experts.

Table 2 and Figure 6 show that most male respondents have answered the survey questions, which can suggest that mostly, male radiologists work in the neuroimaging representations. The males are 14 and the females are 6. Therefore, 70% of males and 30% of females work in the radiology departments.  Figure 7 shows the age frequency for the individual that belongs to different age groups.

Table 3 shows the correlation analysis of the variables entered in the software. The accuracy in critical ML for neuroimaging representation has been considered the dependent variable, and the rest are independent variables. The analysis shows that age is statistically significant with accuracy in CML (Pearson's correlation = 0.792 and *p* < 0.001). Therefore, age has a positive impact on the accuracy of neuroimage representation by 79.2%. However, it does not define that any older age group people will show higher accuracy in ML. To simplify this, the experience in radiology has been determined as well. The experience in radiology has a higher Pearson correlation value (0.812) which suggests that experience in radiology has an 81.2% impact on determining the accuracy of critical ML (*p* < 0.001). Gender does not have any significant relationship with the accuracy of ML in neuroimaging (*p* > 0.1 and Pearson's correlation = 0.219). The years of training in radiology has a statistically significant relationship with the accuracy in ML (*p* < 0.002 and Pearson's correlation = 0.646). Therefore, years of training have a 64.6% impact on accuracy; however, experiences in radiology have an 81.2% impact on ML accuracy. The mean training provided to the ML for neuroimaging representation is for 3.95 years where the relationship between training years and accuracy is weakly significant (*p* > 0.3). This suggests that radiology departments provide approximately 3-4 years of training to the ML where the training does not affect the accuracy. Rather, the accuracy increased with the experience of the radiologists. The correlation value also suggests that accuracy increases with an IQ increase of radiologists (Pearson's correlation = 56.9% and *p* < 0.005). The IQ was determined by a test where the IQ of the radiologists has been identified based on radiology knowledge, and it showed a 56.9% impact on the accuracy.

The ANOVA table also suggests that the entire independent variables are statistically significant (*p* < 0.05) with the dependent variable (Table 4 and Figure 8). Moreover, the *F* value is significantly higher (an *f* value of 3.95 is considered standard). Therefore, it has been interpreted that those experiences in ML and radiology have a strong impact on the accuracy of neuroimaging representation.

Dot plot representation (not shown here) of the correlation between age and ML accuracy in neuroimaging representation suggested that age has a positive impact on the accuracy of critical ML. Dot plot representation of the correlation between radiology experience and ML accuracy suggested that radiology experience has a weak significant relationship with the CML accuracy. Dot plot representation of the correlation between ML training and ML accuracy in neuroimaging representation suggested that both have weak significant relationship with each other.

Lastly, experience in radiology positively impacted the accuracy of critical ML, and training provided to the ML does not have a significant impact on increasing the accuracy. Other graph charts have not been provided as the previous interpretation upheld the outcome vividly.

## 5. Discussion and Findings

The analysis and interpretation suggested that experience in radiology affects ML accuracy positively. The average training years for ML in neuroimage generation and representation are 3-4 in which a standard training duration of ML in radiology is probable. The results showed that training of ML does not have a significant impact on critical ML accuracy. However, the experience of the radiologists has a strong positive impact on critical ML. Abrol et al. suggested that DL is more accurate and advantageous over standard ML where critical ML is similar to this DL [22].

The data from the analysis suggested that the radiology department has standard ML which alone is not enough to improve the accuracy. The experience and IQ of the radiologists improve the neuroimaging representation accuracy [23]. The critical ML here is a critical justification of the ML results by the radiologists. The standard ML might not provide accurate results, and the results need to be justified further by the radiologists for an intelligent decision. Therefore, the final and accurate decision is not dependent on the ML, and critical discussion and justification are required by the professionals [24]. In this regard of standard ML, the authors are suggesting DL approaches along with further training to improve the accuracy [25]. The training can be carried out using the Scikit tool containing large statistical algorithms that will provide a versatile tool for neuroimaging representation [26]. Lanka et al. suggested that fMRI scan images are needed to be simple for classification by the ML [27]. Therefore, the Scikit package of Python is used for the classification and determination of complex images [28] This suggests that a brain MRI scan provides a complex image that cannot be detected accurately by the ML [29]. Hence, an experienced radiologist is required to understand the ML output and to move forward for further decisions. The experienced radiologist is responsible for critically evaluating the ML results, and further decisions will be made (hence named “critical ML” or CML). The CML is not defined by the critical thinking of the machines; however, it defines the critical evaluation by the experts in radiology. The findings suggested that the experiences of radiologists are essential to developing critical ML. The SEM shows how each of the variables impacts each other (Figure 9). SEM suggests that IQ, years of training, and radiology experiences are related to each other which is further related to age. Moreover, the study suggested ML training (learning techniques) and IQ of a radiologist have a positive impact on the accuracy of neuroimaging discrimination [30].

## 6. Conclusion

The study found that critical ML is slightly different from standard ML (SML). Critical ML or CML defined the further evaluation of the SML results by radiologists which will improve the accuracy. Usually, SML provides an output that may not be perfect for making the final decision. Thus, critical thinking is required by radiologists to understand the ML results. The study found that SML cannot determine and evaluate the complex fMRI scanned images accurately. More specifically, the *discriminative nature of SML is not accurate enough* to rely on the decision by the ML only. Thus, an experienced radiologist is necessary to evaluate the ML outputs and that will improve the critical ML accuracy in robust discrimination or neuroimaging representation. It also relies on neural networks to improve the performance of the deep learning network. These approaches are necessary to classify and create different clinical pictures. These images can be used to diagnose a range of neurotic and psychological problems. Some of these networks have to function as human beings, and their performance can go beyond human performance. The integration of traditional neural networks is constantly contributing to the field of neuroimaging research. In addition, SVM's ability to confront nonlinear boundaries with the core mapping method has made it extremely strong in this area. Another popular method that caught the attention of neuroimaging studies in the early 2000s was random forests. In total, ten years of rigorous research was primarily the starting point for the development of this method. In the modern medical system, beneficial effects of ML methods on the generation and detection of various images, especially neurological reflexes, have been observed. A wide range of ML applications can be used extensively to produce neurological images, which will soon increase the clinical development potential. In addition, efficient manipulation and diagnosis of these images can be performed using ML procedures that follow the functions of neural network systems.

## 7. Future Scope

The study in this research has upheld the importance of critical thinking or critical ML (CML) in robust neuroimaging representation. However, CML is based upon the standard ML. Therefore, deep learning (DL) approach can be examined with robust neuroimaging for improving the accuracy. Segmentation and multimodal data can be integrated by other researchers to improve the ML and DL approaches. Other researchers and the current study found that ML cannot predict the output accurately; thus, more research and training are required for leveraging the flexibility of ML.

## Figures and Tables

**Figure 1:** Flowchart of the generation of neuroimages.

**Figure 2:** Graph reflecting the generation of neuroimages through ML [3].

**Figure 3:** Generation of neuroimages with the help of ML approaches [9].

**Figure 4:** Treatment of neurological diseases with the help of ML approaches [11].

**Figure 5:** Fitting of brain-age regressor of a community of aging people [15].

**Figure 6:** Gender frequency showing male respondents are dominating in the radiology department.

**Figure 7:** Age frequency, showing every individual that belongs to different age groups.

**Figure 8:** The probability plot shows the independent variables are closely aggregated with the dependent variable.

**Figure 9:** Structural equation model.

**Table 1:** Descriptive statistics of the samples.

Descriptive statistics			
	Mean	Std. deviation	*N*
Accuracy is critical ML (independent variable)	95.885	2.2408	20
Age	39.00	11.262	20
Gender (1 = male, 2 = female)	1.30	.470	20
Experience in radiology	8.10	5.261	20
Years of training in radiology	3.60	1.046	20
Training provided to the ML algorithms (in years)	3.95	1.731	20
IQ	102.90	7.196	20

**Table 2:** Gender frequency.

Gender (1 = male, 2 = female)					
		Frequency	Per cent	Valid percent	Cumulative percent
Valid	Male	14	70.0	70.0	70.0
	Female	6	30.0	30.0	100.0
	Total	20	100.0	100.0	

**Table 3:** Correlation analysis.

Correlations								
		Accuracy in critical ML [independent variable]	Age	Gender (1 = male, 2 = female)	Experience in radiology	Years of training in radiology	Training provided to the ML algorithms (in years)	IQ
Pearson correlation	Accuracy in critical ML [independent variable]	1.000	.792	.219	.812	.646	.078	.569
	Age	.792	1.000	.358	.895	.826	.073	.576
	Gender (1 = male, 2 = female)	.219	.358	1.000	.200	.364	-.110	.180
	Experience in radiology	.812	.895	.200	1.000	.667	-.051	.677
	Years of training in radiology	.646	.826	.364	.667	1.000	-.012	.323
	Training provided to the ML algorithms (in years)	.078	.073	-.110	-.051	-.012	1.000	-.064
	IQ	.569	.576	.180	.677	.323	-.064	1.000

Sig. (1-tailed)	Accuracy in critical ML (independent variable)	.	.000	.176	.000	.001	.371	.004
	Age	.000	.	.061	.000	.000	.380	.004
	Gender (1 = male, 2 = female)	.176	.061	.	.199	.057	.322	.223
	Experience in radiology	.000	.000	.199	.	.001	.415	.001
	Years of training in radiology	.001	.000	.057	.001	.	.481	.082
	Training provided to the ML algorithms (in years)	.371	.380	.322	.415	.481	.	.395
	IQ	.004	.004	.223	.001	.082	.395	.

**Table 4:** Multiple regression ANOVA output.

ANOVA^a^						
Model		Sum of squares	df	Mean square	*F*	Sig.
1	Regression	66.509	6	11.085	4.987	.007^b^
	Residual	28.896	13	2.223		
	Total	95.406	19			

^a^Dependent variable: accuracy in critical ML (independent variable). ^b^Predictors: (Constant), IQ, training provided to the ML algorithms (in years), gender (1 = male, 2 = female), years of training in radiology, experience in radiology, and age.

## Data Availability

The data shall be made available on request.
